This article has been retracted.

# Clinical Care of Hyperthyroidism Using Wearable Medical Devices in a Medical IoT Scenario

**DOI:** 10.1155/2022/5951326

**Published:** 2022-02-23

**Authors:** Lili Wei, Sujuan Hou, Qiuxia Liu

**Affiliations:** Department of Radiology, Tangshan Gongren Hospital, Tangshan, Hebei 063000, China

## Abstract

This paper presents an in-depth study and analysis of clinical care of patients with hyperthyroidism using wearable medical devices in the context of medical IoT scenarios. According to the use scenario of the gateway and the connectivity of the equipment, the hardware architecture, hardware interfaces, functionality, and performance of the gateway were briefly designed, so as to monitor patients with hyperthyroidism more comprehensively and save labor costs. The gateway can provide access to different devices and adaptation functions to different hardware interfaces and provide hardware support for the subsequent deployment of the proposed new medical communication protocols and related information systems. A medical data convergence information system based on multidevice management and multiprotocol parsing was designed and implemented. The system enables the management and configuration of different medical devices and access to data through the targeted parsing of the underlying medical device communication protocols. The system also provides the automatic adaptation of multiple types of underlying medical device communication protocols and automatic parsing of multiple versions and can provide multiple devices to process fused data streams or device information and data from a single device. The use of event-driven asynchronous communication eliminates the tight dependency on service invocation in the synchronous communication approach. The use of a metadata-based data model structure enables model extensions to accommodate the impact of iterative business requirements on the database structure. Real-time patient physiological data transmission for intraoperative monitoring based on the MQTT protocol and video transmission for intraoperative patient monitoring based on the RTMP protocol were implemented. The development of the intelligent medical monitoring service system was completed, and the system was tested, optimized, and deployed. The functionality and performance of the system were tested, the performance issue of slow query speed was optimized, and the deployment of the project using Docker containers was automated.

## 1. Introduction

Relatively inexpensive domestic infusion monitoring devices have been marketed, but they can only be monitored individually and cannot be networked for systematic management [1]. Clinical infusion work still suffers from untimely fluid replacement, inaccurate infusion speed, and failure to detect infusion failure in time. With the frequent emergence of problems such as inefficient medical treatment caused by the insufficient and unreasonable allocation of total medical and health resources, inadequate medical risk control, weak primary health service system, imperfect medical security system, disorderly production and circulation of drugs and medical equipment, inflated prices, and serious disputes between doctors and patients, the problem of how to solve the “difficulty of seeing a doctor” and “expensiveness of seeing a doctor” caused by the imperfect medical system has become more acute [2]. The development and application of Internet of Things (IoT) technology in the medical field have emerged in the world, such as medical waste tracking management, special patient monitoring management, baby monitoring, and elderly vital signs' home monitoring. As IoT technology has precise sensing ability for mobile individuals, there are numerous mobile devices in the clinical medical field; thus, with the continuous development of IoT technology, it has successfully integrated into the clinical medical industry and has provided great help to the construction of smart therapy, which has now become one of the hot spots that the IoT field is concerned about [3].

A medical examination device with antidropping function for clinical use in hyperthyroidism and its control system includes a central processing and control module, a human body sensing module, an action recognition module, an overflow detection module, a height detection module, a sound alarm module, an opening and closing control module, a drive module, a status indication module, and a power supply module. The present invention can automatically identify human body movements, can realize automatic unpacking, and is convenient for putting the used syringes into the syringe storage box, making the recovery of the syringes convenient and preventing the inspectors from touching the intelligent storage box. For more safety and hygiene, the test tube holder and the intelligent storage box are fixed by the first electromagnet and the second electromagnet, which can make the placement of the test tube holder and the intelligent storage box more stable and prevent them from falling off during use; at the same time, the electromagnetic field is controlled by the control button. The working state of the body is convenient for taking the test tube holder and the intelligent storage box, and the practicability is higher. Cloud computing, big data, artificial intelligence, and so on have been the hot spots of general concern and technical research in various industries in recent years, and their related technologies have gradually become popular and mainstream application technologies in the process of informatization and intelligence in various industries. At the same time, in the medical field, large-scale regional medical and health information systems and large health care data centers are also under construction in full swing [4]. Nursing is an important part of health care delivery, and the application of information technology in nursing can reduce duplication of effort and nursing errors, allowing clinical nursing staff to spend more time caring for patients and substantially improving the quality of nursing services [5]. Therefore, nursing information competence has become a basic quality that every nurse must possess, and the improvement of information technology in medical services is a great driving force for the development of medical care. Through the study of nursing information competence theory and practice, a set of scientific and reasonable evaluation systems of nursing information competence of clinical nursing staff is developed [6]. The index system of nursing information competence of clinical nursing staff can provide an objective reference basis for clinical nursing staff and nursing managers on the one hand, and provide objective reference indicators for cultivating efficient clinical nursing staff and improve the overall information literacy of nursing staff on the other hand [7].

Wireless sensors used in the field of environmental monitoring such as temperature and humidity sensors are widely used in soil monitoring, infrared sensors are widely used in elevator escalator human detection, light sensors and sound sensors are widely used in intelligent electric lights, smoke sensors and flame sensors are widely used in security warning, and so on. These sensors use different networks to upload data and after processing and analysis to achieve real-time monitoring of human health and real-time monitoring of the environment. People from many remote areas flock to cities in search of a better medical environment and resources; especially in many cases, there is a need to ensure high-definition video call capability for ambulances to enable remote preemption. Establishing healthcare information systems that use Internet technology to connect hospitals to hospitals and hospitals to patients can greatly reduce the potential for unnecessary transportation, lodging, travel, and illness delays. However, there are still many shortcomings in the current healthcare information technology. Medical scenarios such as remote video suffer from certain delays due to limitations in network structure and medical informatics equipment. At the same time, there is a wide variety of medical informatics, which needs to be optimized for specific medical informatics scenarios.

## 2. Related Work

This section discusses the specific implementation of the Internet of Things in the health field and proposes a construction concept related to the smart hospital based on the Internet of Things [8]. It is considered that smart medicine is a medical system that combines electronic medical records, electronic health records, and medical Internet of Things with medical cloud data as the core and Internet of Things and data transmission and exchange as the technology to build medical and health services and optimal management [9]. Based on the new medical and health service model of “Internet + health care,” the shortcomings of the traditional medical service model are analyzed, and the tasks of intelligent medical action are proposed, mainly including medical Informa ionization and medical body construction [3]. The construction of smart medical applications based on IoT technology, including mobile medical care, medical equipment management, and smart hospital service system, was elaborated to gradually realize the combination of IoT and medical services [10]. The purpose of cancer treatment is not only to prolong survival time but also to maintain and improve the quality of survival, which is not only in line with the natural law of cancer development but also consistent with the humanistic concept of “people-oriented” advocated by the state [11]. The evaluation of the quality of survival of cancer patients has become an important aspect of cancer care, but previously it mainly focused on common tumors such as gastric cancer, lung cancer, and breast cancer [12].

Since the incidence of thyroid cancer has shown a trend of increasing year by year in recent years and at the same time, with the advancement of medical screening, diagnosis, and treatment techniques, the postoperative survival of thyroid cancer is more considerable, many scholars have begun to focus on the study of the survival quality of thyroid cancer patients [13]. Medical process monitoring usually still uses manual rounds, transcription of infusion orders, and transcription of inpatient information small card, so the hospital ward nurses also need to blindly run back and forth between the nurse's station and the ward and cannot have a clear sense of the patient's various help but make the planning of the nurses work greatly reduced [14]. With the continuous development of smart mobile devices, mHealth has also begun to influence the way of medical management, doctor-patient communication mode, and health product innovation. Medical services and information are provided using computers, handheld mobile terminals, and software for smart devices combined with mobile communication technology connected to the network [15]. Later, as mobile communication technology continues to develop, increased hospitals are building mobile health care workstations using mobile devices such as PDAs.

The traditional infusion set is still the most used infusion tool in clinical care, and its monitoring method is based on manual inspection. During infusion, the bag or bottle is hung above the needle insertion site of the infuser, and the drip rate is set by the nurse according to experience by manually adjusting the pulley on the infusion tube. When the infusion is about to end or when discomfort occurs during the infusion, the patient or caregiver is required to manually notify the health care worker to come and deal with it in time. This not only increases the labor intensity of health care workers but also makes clinical safety not improved. The management system monitors the infusion status in real time in the field through wireless communication technology, calculates the end time of infusion, and gives an alarm to remind us when the infusion is finished. Any special situation during infusion can be contacted with the nurse main console through the patient call interconnection system. The system can not only reduce the labor intensity of nursing staff and improve work efficiency but also significantly reduce the hidden dangers that may occur during the infusion process, which is the future application trend of clinical medical nursing work.

## 3. Analysis of Clinical Care of Hyperthyroidism with IoT Wearable Medical Devices

### 3.1. Medical IoT for Wearable Medical Devices Design

The medical scenario considered in this paper is the scenario where multiple medical devices need to be connected and provide real-time monitoring to the patient, such as an operating room or emergency ward. In existing medical scenarios, it is often necessary to add multiple medical monitoring devices such as monitors, ventilators, and syringe pumps. In addition to this, there are also environmental monitoring devices such as cameras, monitor video encoding boxes, and environmental sensors. All these devices need to be set up independently on the device by the healthcare provider; for example, the monitor needs to be set up for network settings, IP settings, data display item settings, alarm settings, and so on, the syringe pump needs to be set up for push mode, drug settings, channel settings, alarm settings, and so on, the ventilator needs to be set up for ventilation mode, respiratory rate, airway pressure, tidal volume, alarm settings, and so on, and the camera and coding box need to be logged into the device access page for resolution, bit rate, push stream address settings, and so on.

At the same time, the medical process also requires medical personnel to always monitor the operating status of the equipment and alarm information to prevent medical accidents caused by unexpected equipment failures and parameter alarms. In addition, the maintenance of equipment also poses certain difficulties; after the failure of medical equipment, medical staff often need to consult the equipment manufacturer or hospital technicians to recover according to the equipment manual [16]. Environmental monitoring devices such as cameras also require login to the device page to enter a user name, password, and device IP before they can be accessed, as does the setup of the coding box.

At the same time, the unified management of devices such as device registration, device online, and device offline also needs the uniqueness of the device identification to be distinguished, how to ensure the uniqueness of the device is also a problem that needs to be studied, and a more reliable scheme is based on the device address (MAC address, USB address, and serial port address) and device protocol to register the device ID as shown in Figure 1.

There is more overlap in the way these three models apply IoT, and the main component of the project lies in the information system. Existing IoT products are mostly designed to solve specific challenges and hardly meet the needs of most healthcare organizations for system functionality. The deep integration and scale utilization of IoT and healthcare require a mature all-in-one applicable solution.

This paper examines the impact of IoT on the development of medical consortia on a macrolevel. There are various forms of IoT applications, which are currently divided into four categories, care management, medical device management, supply management, and wearable devices, and different applications have different impacts on medical consortia, while medical consortia are divided into four categories, medical groups, medical communities, specialty alliances, and remote collaboration networks, and different medical consortia have different needs for IoT [17]. So microscopic impact of IoT on the development of medical consortia is governed by the form of IoT and the type of medical consortia. In contrast, the study of the macroimpact is not influenced by these factors. In terms of aiding decision-making, the scores of macroimpact are categorized based on factors such as application technology and type of IoT project, and the conclusions of the analysis can be better used as a basis for decision-making. A neural network algorithm is used because our experimental data are limited, and only the algorithm using a neural network can get better results.

The ward call system is a comprehensive system project, which should be considered from various aspects such as its function, performance, cost, and application of modern related technology. Based on such requirements, it is suitable to develop an integrated intelligent medical call system that integrates the functions of bed call, bathroom call, and corridor screen display using CAN bus technology, as shown in Figure 2. As ZigBee technology itself is suitable for wireless data transmission in a small area, in an environment with a large area and relatively complex building structure such as a hospital ward, the loss rate of wireless signals is inevitably high; if the data reception and forwarding capacity are increased by adding terminals, the problems of wireless signal collision and high probability of error codes cannot be solved; it is impossible to set up a large sensing network covering the whole hospital. It is impossible to set up a large sensor network covering the whole hospital.

The ZigBee terminals are wired and powered because they need to forward signals at any time and have high energy requirements. The ward call system uses the CAN bus for data transmission, which is mainly based on security considerations to ensure reliable transmission, but there are disadvantages such as poor system scalability and the need for wiring in the ward.

Any unit connected to the bus can start sending messages if the bus is idle, and if two or more units on the bus start sending messages at the same time, the priority can be determined by receiving or blocking the message according to its ID (identifier). In the ward call system, the call button located in the ward only needs to be pressed when the patient has an emergency to send a call message to contact the nurse and does not transmit the message at all times. The number of nodes that can be connected to the CAN bus is theoretically unlimited, but it is limited by the bus time delay and load capacity. If the number of connected nodes needs to be increased, then the communication speed can be reduced; conversely, if the transmission speed needs to be increased, then the number of connected nodes can be reduced.

For the award, the number of wards is relatively high. The main functions of the clinical medical information management system are to monitor the infusion status of patients in real time, to respond to patients' needs in time, to understand the situation and needs of each ward, and to realize scientific management of the whole ward and ward so that the efficiency of medical and nursing workers can be improved, the overall service quality of the hospital can be improved, and the medical safety and patient satisfaction can be enhanced.

### 3.2. Analysis of Clinical Care in Hyperthyroidism

With the continuous development of business, the amount of code of the whole system will become increasingly complex, and the system architecture will become increasingly complex. There are many problems faced by using monolithic architecture, such as low development efficiency, increasing maintenance cost, large deployment impact, poor scalability, and high technology selection cost. Therefore, at the beginning of the system design, the system should be split into multiple modules with the idea of microservices [18]. When the system is gradually upgraded with iterations, the vertical expansion of the system can be achieved by upgrading the in-service functionality of individual services. When the upgrade of existing microservices cannot meet the business needs of the system, new microservices can be added to provide new service capabilities to cope with complex business needs.

(1) $$\begin{array}{c} R_{1}=\frac{V_{cc}^{2}-V_{F}^{2}}{I_{F}^{2}}. \end{array}$$

In the formula (1), *R*_1_ represents the serial number 1 resistance, *V*_*cc*_^2^ represents the voltage difference, *V*_*F*_^2^ represents the negative voltage, and *I*_*F*_^2^ represents the current of the circuit. The way services communicate with each other also affects the degree of interdependence of the services. Synchronous and asynchronous communication are two ways to implement messaging between services. Rest HTTP is a request/response-based synchronous invocation method of communication that encapsulates parameters into JSON format for messaging. Although this communication method is simple to invoke, one party sends a request and waits for the request to be transmitted to the other party and waits until the other party returns after the request has been fully processed before proceeding to the next operation.

Another way of communication between services is asynchronous message invocation, and the message sender only needs to send the message and does not need to care which service is to receive this message; that is, the service does not know who they are called by and does not know which service they will call. Detaching the entire flow of business execution from the module reduces the coupling between the caller and the called, as shown in Figure 3.

It provides edge computing platform services, including support for edge application deployment, providing a unified portal for application deployment. It supports configuration distribution with streaming media equipment, and reports streaming configuration information to the dedicated network operation management platform. It also supportsthe provision of service capabilities, including location services, bandwidth management services, and wireless network information to industry applications through the wireless side or core network side interface. Based on specific business scenarios, it supports providing applications with capabilities such as video streaming and AI algorithm library to meet application requirements.

The scheduler can be seen as a parent node, and the queues/schedulers being scheduled are seen as children. The scheduler can schedule multiple queues and can schedule multiple schedulers. The parent node is the traffic convergence point for multiple child nodes. The classification rules of nodes at different levels can be oriented to different classification needs (e.g., users and business types), each node can specify classification rules and control parameters to classify and control the traffic once, and different control actions can be done on the traffic at different nodes, thus realizing multiservice, multilevel, and multiuser management of the traffic.

(2) $$\begin{array}{c} \frac{R_{11}}{R_{10}-R_{11}}\cdot V_{cc}=1000mV, \end{array}$$

(3) $$\begin{array}{c} R_{10}\approx 8R_{11}. \end{array}$$

In the formula (2), *R*_11_ represents the resistance between 1 and 2, *R*_10_ represents the resistance from the initial point to point 1, and the voltage value difference is 1000 mV. First, the subject of assessing the impact of IoT on the development of healthcare clusters is one or more healthcare clusters, with more than ten healthcare organizations in each cluster, and it is practical to use success rates as impact evaluation. Second, the market size in the field of medical IoT has maintained a 25% growth rate in 10 years and is forecast to remain the same in five years. Therefore, the proportion of IoT projects and the future changes in the development trend are not significant.

(4) $$\begin{array}{c} M\left(x\right)=w_{2}\sigma \left(w_{1}x\right), \end{array}$$

where *M*(*x*) represents the state at the *X* position, *w*_2_ represents the weight of the second point, *σ* represents the state coefficient, *w*_1_ represents the weight of the first point, and *x* represents the corresponding position. For IoT projects with high technology, the breakthrough products make a certain impact indicator score of 1, but the overall score tends to be close to 0 due to the difference in technology or application focus of other IoT projects. But because IoT technology is in the overall development stage, the overall change in the impact of IoT on healthcare in the next five years is small, and the impact of high technology projects, although growing faster, will not affect the overall statistical level as shown in Figure 4.

Firstly, based on the author's source, the data source, and the type of IoT projects, applied IoT technologies were counted, and percentage stacked bar graphs were plotted to understand the researcher's preference. After analysis, the researchers showed differences in the source of data and the two IoT technologies applied. Researchers from hospitals and schools were more likely to evaluate the impact of IoT on the development of healthcare clusters through qualitative methods, while researchers from the health sector and businesses were more likely to evaluate through case effects. Researchers from hospitals are mainly users of IoT products, researchers from schools are mostly product development designers, and the evaluation of the effects of IoT applications by these two types of researchers is more subjective. The technologies applied by researchers from hospitals and schools are mainly wearable devices, while health authorities and companies focus more on the integrated use of IoT technologies [6]. From Figure 4, it is known that researchers from schools and hospitals together account for 72.9% of the total researchers, so researchers from hospitals and schools will have more influence in the evaluation of the impact of wearable device cases on the development of health care clusters.

(5) $$\begin{array}{c} Q_{N}\left(w\right)=\frac{1}{2}\sum_{i,j}{\left(1+P_{ij}\right)}^{2}\left(m_{i}-m_{j}\right). \end{array}$$

In formula (5), *Q*_*N*_(*w*) represents the state where the weight is *w* at the position of *N*, *P*_*ij*_ represents the weight component of the *i*-th row and *j*-th column, *m*_*j*_ represents the initial component, and *m*_*i*_ represents the end component [19]. The lack of interoperability of medical information systems has always been an important factor constraining the construction of health informatization, and there are two reasons for the difficulty in sharing information [20].

The study on the working status of the study subjects found that 53 cases (30.64%) were currently engaged in domestic work and 44 cases (25.43%) were still working, which was related to the fact that the survey subjects were mostly middle-aged women mainly from rural areas. The types of medical insurance of the survey respondents were mainly new rural cooperative medical insurance and urban employees, with 91 cases and 62 cases, accounting for 52.60% and 35.84%, respectively [8, 21, 22].

## 4. Analysis of Results

### 4.1. Performance of Medical IoT Systems for Wearable Medical Devices

As multiple surgeries are performed at the same time in a hospital, multiple monitoring devices are used to monitor the physiological status of the patient during each surgery. The real-time data transmitted from the gateway to the upper layer during the surgery includes both the physiological data of the patient collected by the monitoring device and the alarm information of the monitoring device. In addition to this, the client may also downlink the configuration information of the device at this time, so the concurrency of real-time data information received by the client at the same moment can be large. Using multiple threads to receive the patient's physiological data, alarm information, and configuration information separately, and using multiple threads to process the real-time data information, the CPU resource utilization can improve.

Considering that each time the real-time data arrives, a thread needs to be created to process the data, and after processing is complete, the thread must be destroyed to avoid resource usage; this process will keep consuming CPU resources, so a thread pool is used to implement a thread reuse mechanism and eventually interthread scheduling. The real-time curve board for ventilators and syringe pumps is designed according to the real screen of ventilator and syringe pump devices, and the expansion capability is reserved here to switch the display of different content on the page to accommodate the display of content for other types of device access. The real-time data display for the monitor is shown in Figure 5.

A complete test environment is set up in the laboratory as shown in Figure 5. The gateway communicates with the medical devices through the default intranet IP in the gateway, and the gateway, video encoding box, and network pushing camera are then connected to the laboratory LAN to achieve data and video transmission; the server and client are connected to the laboratory LAN to achieve system access and data communication with the gateway. The hardware environment is mainly a monitor connected to the gateway through the network port, a ventilator connected to the gateway through the serial port, and a syringe pump connected to the gateway through the USB port. Real-time data are collected by these three devices and collected by the gateway, and then the gateway connects to the lab intranet through a wireless connection to realize data transmission with the server.

The video encoding box is connected to the monitor through a VGA port to collect the live video stream of the screen and then connected to the router through the network port to realize the live stream push. The webcam collects indoor scenes and connects to the router through the network port to realize the live streaming push of indoor scenes.

The operation functions of user management are routine operations, so there is no need to consider the concurrency problem, and only the feasibility of the function needs to be tested, as shown in Figure 6. The operation management module can complete the basic operation of the operation room and can realize the basic functions of intraoperative monitoring, which can enter the operation room to view the scene of the operation, perform the operation triggered by the key time points of the operation process, view the monitoring records and quality control records, view the live screen of the monitor screen and the live video broadcast of the scene captured by the camera, and view the real-time collected parameters of the anesthesia machine, the parameters of the syringe pump, the monitor parameters, and so on, and the basic functions of intraoperative monitoring can be achieved normally by changing different models of test devices during testing.

As the underlying gateway realizes the adaptation to different types of medical devices, the data collected by the devices are parsed and processed into a unified format and then sent to the server, and the gateway can realize the transmission of real-time data, so when the data are transmitted to the server, the differences between devices of different manufacturers are already shielded. The gateway and device management module realize the unified control of the gateway and various medical devices, and the system supports the management of various types of medical devices. Alarm management realizes the management of medical device alarms and abnormal alarms of physiological indicators of patients during surgery. In summary, the overall system function test pass rate is 100%, which means that all the modules of the system can be realized normally, and the system is currently applicable to all the gateways that have been successfully adapted to the devices.

### 4.2. Clinical Care Outcomes in Hyperthyroidism

Informatization of nursing services not only enhances efficiency and allows nursing staff to spend more time facing patients but also leads to higher patient satisfaction with the nursing staff. Therefore, the integration of healthcare services with Internet platforms is becoming the direction of information technology development in medium and large hospitals. Nursing staff plays an important role in hospitals, while some of our nursing staff have not yet been able to acquire some knowledge and skills in nursing informatics. As nursing staff should all need to master the professional knowledge and application related to nursing informatics as well as have the ethics related to nursing informatics.

It was concluded from reviewing a large amount of literature that the evaluation system of nursing information competency in China is necessary because it is less and one-sided compared to foreign studies. The nursing information competence evaluation index system established in this study can provide a theoretical basis for the development of a scientific and reasonable nursing informatics training program for nursing staff. The increasing number of hospitals applying 5G “Internet medicine” shows the importance of establishing a set of nursing informatics evaluation systems suitable for clinical nursing staff. The development of nursing informatics education and the improvement of nursing informatics personnel are effective means to reduce nursing errors and improve work, as shown in Table 1.

This study illustrates that the process of information technology construction must put the legality and security of information in the first place, information security is a prerequisite for the behavior of nursing information technology, and it is urgent to improve the awareness of information security of nursing staff; if there are information security problems, all information construction will be impossible to talk about, so it is necessary to first guarantee the security of nursing information and establish a security barrier to prevent nursing errors and management Vulnerability. The second level indicator is “nursing informatics awareness,” and the weight coefficient of nursing staff's “subject awareness” is 0.1295, which indicates that nursing staff needs to constantly realize that they need to continuously learn to make up.

This indicates that nursing staff needs to be aware of the need for continuous learning to make up for their shortcomings, improve nursing information capabilities to enhance work efficiency, and realize the organic integration of information technology with nursing work and nursing management. “Knowledge of nursing informatics” has a low weighting factor compared with other indicators, but it is indispensable in nursing work. Without mastering the concepts, views, and theoretical systems of relevant theories and without a certain amount of relevant theoretical training, it is impossible to put forward any new views and concepts even if the practice time is longer and the practice is more, let alone put forward systemic new theories.

However, considering that all patients were aware of their thyroid ultrasound results before admission and with the increasing accuracy of medical technology, patients had a basic judgment of their condition before surgery; coupled with the health education of the medical staff, they had a scientific understanding of the good prognosis of thyroid cancer, as shown in Figure 7.

Knowledge of thyroid cancer disease is extremely low, and people fail to realize the closeness of these factors to the prognosis of the disease. Finally, the reason for the lack of statistically significant knowledge about the pathology of the disease may be related to the fact that some of the patients have postoperative pathological results of thyroid cancer, although their family members concealed the true nature of their pathology, considering that all patients knew the results of their thyroid ultrasound before admission, and with the continuous progress of medical technology ultrasound results becoming more and more accurate, patients have a basic judgment of their condition before surgery.

In life, the role of women is multiple; on the one hand, like men, they bear the important responsibility of promoting social development, and on the other hand, they also bear the sacred responsibility of taking care of their families and giving birth to and educating their offspring; at the same time, women have special body structure and physiological mechanism; therefore, the physical and mental health of women will be directly related to the harmony of a family or even the whole society. Strengthening the psychological care of female thyroid cancer patients will help to reduce the occurrence of anxiety, improve the quality of survival, and promote the prognosis of the disease.

## 5. Conclusion

In this paper, a new medical-oriented IoT gateway is proposed for the traditional medical scenario where the underlying medical devices are of various types and the data communication protocols used are closed to each other, the data cannot be processed and aggregated effectively, and the hardware, interface communication protocols, and information system of the gateway are designed and implemented. The gateway can provide a variety of hardware interfaces for device access and is equipped with a high-capacity lithium battery to cope with emergency emergencies. The internal information system can parse the protocols of the underlying medical devices that access the gateway to obtain medical monitoring data, and the interface communication protocol can provide data access interfaces and medical device management interfaces to external terminals. Therefore, the gateway can unify the management and configuration of all medical devices and IoT devices in the ward, automatically resolve the medical protocols of the underlying medical devices to obtain data, and realize the real-time pushing of data streams through the processing and fusion of data. By deploying the gateway in a hospital operating room for field testing, it is found that the gateway can effectively shield the differences of the underlying devices in the ward, the diversity of medical communication protocols, and the isolation of data and realize the unified management and configuration of devices, the automatic parsing of medical communication protocols, the secure encryption of data processing and fusion, and the real-time pushing of monitoring data of multiple devices in the ward. The relevant functions of the gateway have been effectively verified, and good remote real-time monitoring has been achieved. Our research results can be fully applied in practical situations.

## Figures and Tables

**Figure 1:** Medical IoT framework for wearable medical devices.

**Figure 2:** Signal transmission diagram of the call system.

**Figure 3:** Status of quality of survival.

**Figure 4:** Proportion of data sources.

**Figure 5:** Real-time data display of the monitor.

**Figure 6:** Graph of test results.

**Figure 7:** Outcome of care.

**Table 1:** Multiple linear regression analysis.

Independent variable	B	Beta	FA	P
Constant	0.892	0.617	0.732	0.694
Hospital level	0.484	0.939	0.598	0.769
Does the hospital have	0.736	0.512	0.603	0.766
Information equipment	0.984	0.764	0.601	0.443

## Data Availability

The data used to support the findings of this study are available from the corresponding author upon request.
